# Safety and Efficacy of Early Carotid Endarterectomy in Patients with Symptomatic Carotid Artery Stenosis: A Meta-Analysis

This article has been retracted.

**DOI:** 10.1155/2021/6623426

**Published:** 2021-01-08

**Authors:** Xiao Chen, Jing Su, Guojun Wang, Han Zhao, Shizhong Zhang, Tao Liu, Xindi Su, Ning Zhou

**Affiliations:** ^1^Shandong First Medical University (Shandong Academy of Medical Sciences), Jinan City, Shandong Province, China; ^2^Shandong Taian City Central Hospital, Taian City, Shandong Province, China; ^3^Jinzhou Medical University, Jinzhou City, Liaoning Province, China; ^4^Shandong Taian City Central Hospital Branch, Taian City, Shandong Province, China

## Abstract

**Design:**

A systematic document retrieval of studies published in the past 10 years reporting periprocedural stroke/mortality/MI after carotid endarterectomy (CEA) related to the time between CEA and qualifying neurological symptoms. The application database has “PubMed, EMbase and Cochrane databases.” RevMan5.3 software provided by the Cochrane collaboration was used for meta-analysis.

**Results:**

A systematic literature search was conducted in databases. A total of 10 articles were included in this study. They were divided into early CEA and delayed CEA with operation within 48 h, 1 w, or 2 w after onset of neurological symptoms. Incidence of the postoperative stroke in patients undergoing delayed CEA (≥48 h) was significantly higher than patients with delayed CEA (<48 h) (OR = 2.14, 95% CI: 1.43-3.21, *P* = 0.0002). The postoperative mortality of patients after delayed CEA (≥48 h) was significantly higher than patients after early CEA (<48 h) (OR = 1.35, 95% CI: 1.06-1.71, *P* = 0.02). The risk of postoperative mortality of patients treated with delayed CEA (≥7 d) was significantly higher than patients after the early CEA group (<7 d) (OR = 1.69, 95% CI: 1.21-2.32, *P* = 0.001).

**Conclusion:**

Early CEA is safe and effective for a part of patients with symptomatic carotid stenosis, but a comprehensive preoperative evaluation of patients with carotid stenosis must be performed.

## 1. Introduction

Stroke represents the fourth cause of death worldwide; carotid artery stenosis is one of the important causes of stroke [1]. Carotid endarterectomy (CEA) has been identified as the preferred treatment for carotid stenosis. In the past, it was believed that the risk of early recurrent TIA or stroke after the onset of neurological symptoms is not high, so CEA should be delayed for at least 6 weeks after an onset of neurological symptoms, and operating early on a recently symptomatic “unstable” carotid plaque was associated with an increased risk of perioperative stroke [2]. In recent years, early surgical intervention within 1-2 weeks of symptom onset has been advocated for patients with symptomatic carotid artery stenosis [3]. Therefore, the timing of CEA surgery has been gradually attracted the attention of all, and studies on it have also increased gradually in recent years. The current recommendations about when to perform carotid endarterectomy to patients with sCAS rely on multiple uncertainties. The present study reviewed the studies published in the past 10 years, and the risks of postoperative complications of early CEA or delayed CEA were summarized, and meta-analysis was made.

## 2. Methods

A systematic literature search was conducted in PubMed, MEDLINE, Embase, and Cochrane databases. The retrieval language is English. Various synonyms and related Medical Subject Headings (MeSH) for “carotid artery,” “operation timing,” “early endarterectomy,” “delayed endarterectomy,” “carotid stenosis,” “Endarterectomy, Carotid” to build the search syntax.

### 2.1. Inclusion Criteria and Study Endpoints

Inclusion criteria: (1) patients with symptomatic carotid stenosis; (2) the treatment was carotid endarterectomy; (3) patients were grouped according to symptom timing of surgery. Articles were excluded if they were (1) noncontrolled test, (2) did not study human subjects, and (3) not published in full text. If clinical studies were conducted by the same team, the articles with the most complete data, the largest sample size, or the most relevant results are selected.

The primary endpoints were stroke and mortality after CEA. The secondary end point was MI. They were divided into early CEA and delayed CEA with operation within 48 h, 1 w, or 2 w after onset of neurological symptoms.

### 2.2. Study Selection and Data Extraction

Three independent investigators comprehensively evaluated the included articles, carefully read the abstract of the articles, and evaluated the eligibility based on the full text, and judgement differences were resolved by communicating with each other. References of the included articles were carefully examined and searched for some references if necessary. Data of the included articles were recorded on a spreadsheet, including the basic characteristic of the paper (year of publication, author, research method, etc.), the year of recruitment of patients; baseline characteristic of preoperative patients, grouped base on CEA timing, postoperative complications, etc. If some studies do not report relevant data, corresponding authors were requested to provide these data. If the authors are still not provided, they will be excluded in some outcomes or subgroup group. Although we tried to contact the authors to refine the study, we did not obtain unpublished data.

### 2.3. Assessment of Risk of Bias and Methodological Quality

Assessment of risk of bias according to the Newcastle-Ottawa quality assessment scale. Evaluation standard: (1) Is the case definition adequate?; (2) Representativeness of the cases; (3) Selection of Controls; (4) Definition of Controls; (5) Comparability of cases and controls on the basis of the design or analysis; (6) Ascertainment of exposure; (7) Same method of ascertainment for cases and controls; (8) Nonresponse rate.

### 2.4. Statistical Analysis

If more than 1 study had available data, and it will be performed and analyzed, an *I*^2^ value was calculated to describe the percentage variance among studies attributable to heterogeneity. All meta-analyses were conducted using Review Manager (RevMan version 5.3). For each binary variable, an odds ratio (OR) and 95% confidence intervals (95% CI) were used to compare early CEA and delay CEA. *I*^2^ value was used to estimate the degree of heterogeneity, *I*^2^ values ranging from 0% to 100% (0-24%, low heterogeneity; 25-49%, moderate heterogeneity; 50%-74%, high heterogeneity; 75-100%, extreme heterogeneity). When there is low heterogeneity value (*I*^2^ ≤ 25%), Mantel-Haenszel fixed effect model was used for data synthesis. When there is high heterogeneity value (*I*^2^ > 25%), the Mantel-Haenszel random effect model was selected as the endpoint, and sensitivity analysis was conducted to find the source of heterogeneity. *P* values were calculated for all subgroups. When *P* < 0.05, there was a statistical difference; otherwise, there was no statistical difference.

## 3. Results

### 3.1. Search Results

We used keywords to detect 377 related articles in each database and excluded 48 duplicates removed. A total of 95 articles were selected to check the full text by reading basic information and abstracts. The remaining 22 articles after excluding 73 articles according to asymptomatic patients, operation timing, and no reporting data were required. Finally, 10 articles were included for analysis (Figure 1).

### 3.2. Quality Assessment

The quality of the included studies was adequate, all of them have been published for nearly 10 years, and a total of 29,457 patients were included (Table 1). Quality evaluation was conducted according to the Newcastle-Ottawa quality assessment scale (Figure 2).

### 3.3. Outcomes

Stroke analysis of seven studies revealed that patients with delayed CEA (>48 h) had a higher incidence of postoperative stroke than those with early CEA (≤48 h) (OR = 2.14, 95% CI: 1.43-3.21, *P* = 0.0002); Analysis of seven studies revealed that there was no statistically significant difference in the incidence of postoperative stroke between delayed CEA (>1 w) and early CEA (≤1 w) (OR = 1.37, 95% CI; 0.97-1.92, *P* = 0.07); Analysis of eight studies revealed that there was no statistically significant difference in the incidence of postoperative stroke between delayed CEA (>2 w) and early CEA (≤2 w) (OR = 1.07, 95% CI: 0.77-1.49, *P* = 0.69).

Analysis of this group revealed the incidence of postoperative stroke in patients with delayed CEA was significantly higher than that of patients with early CEA (OR = 1.37, 95% CI: 1.11-1.69, *P* = 0.003) (Figure 3).

Mortality analysis of six studies revealed that patients with delayed CEA (>48 h) had a higher incidence of postoperative mortality than those with early CEA (≤48 h) (OR = 1.35, 95% CI: 1.06-1.71, *P* = 0.02). Analysis of five studies revealed that patients with delayed CEA (>1 w) had a higher incidence of postoperative mortality than those with early CEA (≤1 w) (OR = 1.69, 95% CI: 1.24-2.32, *P* = 0.001). Analysis of seven studies revealed that there was no statistically significant difference in the incidence of postoperative stroke between delayed CEA (>2 w) and early CEA (≤2 w) (OR = 0.89, 95% CI: 0.51-1.55, *P* = 0.67).

Analysis of this group revealed that the incidence of postoperative mortality in patients with delayed CEA was significantly higher than that of patients with early CEA (OR = 1.41, 95% CI: 1.17-1.68.69, *P* = 0.0002) (Figure 4).

Myocardial infarction analysis of seven studies revealed that there was no statistically significant difference in the incidence of postoperative MI between delayed CEA and early CEA, whether it has 1 w (OR = 2.5, 95% CI: 0.38-16.50, *P* = 0.34) or 2 w (OR = 1.33, 95% CI: 0.2-8.69, *P* = 0.76) (Figure 5).

Analysis of this group revealed that there was no statistically significant difference in the incidence of postoperative MI between delayed CEA and early CEA (OR = 1.81, 95% CI: 0.48-6.8, *P* = 0.38).

### 3.4. Publication Bias

It can be seen that the overall bias is acceptable by drawing the funnel plot (Figure 6). If the heterogeneity of the results is too high (*I*^2^ > 25%), sensitivity analysis will be used to find the source of heterogeneity and remove it after it is identified.

## 4. Discussion

CEA is an effective method to treat patients with symptomatic carotid artery stenosis. The choice of surgical timing is closely related to the patient's postoperative recovery. The views on the timing of CEA to treat patients with sCAS have been changed with the development of CEA and perioperative management techniques. The traditional view of carotid revascularization was the intervention is delayed by at least six weeks after an acute stroke. The studies published in the 1960s and 1970s suggested that patients with ischemic stroke after early intervention have a higher risk of postoperative cerebral hemorrhage [14]. At that time, a retrospective study showed that the perioperative outcomes of patients with sCAS after early CEA were generally worse than delay CEA [15, 16].

However, a growing number of studies have found that early CEA may be associated with a slightly higher risk of perioperative complications in recent years, but it still is the best chance for symptomatic patients to avoid future strokes [17, 18]. The results of subgroup analysis of NASCET [19, 20] showed that the earlier CEA was performed after onset of neurological symptoms (TIA or minor stroke), the more significant of the prevention effect of secondary stroke in patients. A large number of evidences [17, 20, 21] revealed the safety of early CEA within 1-2 weeks after onset of a TIA or minor stroke. Dorigo et al. [21] indicate that CEA was performed within 15 days after onset of TIA or stroke, and risk of the perioperative stroke was <3.5%. The present study revealed that the incidence of postoperative stroke in patients with delay CEA was significantly higher than that of patients with early CEA (OR = 1.37, 95% CI: 1.11-1.69, *P* = 0.003); the incidence of postoperative mortality in patients with delay CEA was significantly higher than that of patients with early CEA (OR = 1.41, 95% CI: 1.17-1.68.69, *P* = 0.0002). These outcomes may indicate that it is safe and effective of early CEA for a part of patients with sCAS. But it should be noted that the selection of early CEA or delay CEA for patients must be careful according to the current study. Ballotta et al. [22] categorize patients according to the Rankin assessment scale, Rankin 0/2 indicated minor or nondisabling stroke, and Rankin 3/5 defined major or disabling stroke; the study showed early CEA after a nondisabling ischemic stroke can be performed safely. Capoccia et al. [23] suggest that minimizing the time for intervention for patients National Institutes of Health Stroke Scale (NIHSS) ≥8 not only reduces the risk of recurrence but can also improve neurologic outcome. Therefore, the timing of the operation should be based on a comprehensive assessment of the patient.

The present study revealed that there was no statistically significant difference in the incidence of postoperative MI between delayed CEA and early CEA. Roussopoulou et al.'s [24] findings highlight that urgent CEA performed within two days from the index event is related to a nonsignificant increase in the risk of periprocedural MI, this is the same as the results of our study. Early CEA might not increase the risk of postoperative MI.

### 4.1. Limitations

CEA has been used for many years, and the perioperative management and operative style are generally uniform. Most of the articles are recorded, but some are not mentioned. It is not clear whether some patients are used technologies such as pCEA, etc. The follow-up time of the 10 articles that were included in the study was not the same; however, most of them could be followed up more than 30 days; the longest follow-up time could be up to 10 years. There is no clear data about the perioperative medication treatment of CEA. Symptomatic carotid artery is now not graded on admission. Patient with sCAS is not classified.

## 5. Conclusions

Early CEA is safe and effective for a part of patients with symptomatic carotid stenosis. Early CEA may be able to reduce postoperative complications of patients with sCAS, but a comprehensive preoperative evaluation of patients with sCAS must be performed. The safety of early CEA requires further evaluation in larger datasets.

## Figures and Tables

**Figure 1:** Flowchart showing the selection of articles for review.

**Figure 2:** Assessment of risk of bias and methodological quality.

**Figure 3:** Differences in the incidence of post-CEA stroke between the early CEA groups and delayed CEA.

**Figure 4:** Differences in the incidence of post-CEA mortality between the early CEA groups and delayed CEA.

**Figure 5:** Differences in the incidence of post-CEA myocardial infarction between the early CEA groups and delayed CEA.

**Figure 6:** Funnel plot.

**Table 1:** Baseline characteristics of the included studies.

Trial	Year		Study size	Design	Operation timing	Outcome
	Publication	Recruitment				
Annambhotla et al. [4]	2012	1999-2010	312	Retrospective cohort study	0-7 d; 8-14 d; 15-21 d; 22-30 d; >30 d	Mortality/MI/stroke
Kjorstad et al. [5]	2017	2014-2015	371	Prospective	0-2 d; 3-7 d; 8-14 d; >14	Mortality/stroke
Rantner et al. [6]	2015	2004-2013	761	Retrospectively cohort study	0-2 d; 3-7 d; 8-14 d	MI/stroke
Stromberg et al. [7]	2011	2008-2011	2596	Prospectively	0-2 d; 3-7 d; 8-14 d; >14	Mortality/stroke
Salem et al. [8]	2012	2008-2010	109	Prospective	1-7 d; 8-14 d	Mortality/MI
Tsantilas et al. [9]	2017	2004-2014	401	Prospectively	0-2 d; 3-7 d; 8-14 d; >14	Mortality/stroke/MI
Ferrero et al. [10]	2010	2004-2007	285	Retrospective cohort study	<48 h; 48 h-2 weeks; 2-4 weeks; 4-8 weeks; 8-24 weeks.	Mortality/stroke/TIA
Villwock et al. [11]	2014	2002-2011	23729	Retrospective cohort study	Within 2weeks	Mortality/stroke
Nordanstig et al. [12]	2017	2010-2015	418	Prospectively	48 h; 48 h-2 w	Stroke/TIA
Sharpe et al. [13]	2013	2008-2013	475	Retrospective cohort study	2 d; 3-7 d; 8-14 d; >14 d	Stroke/TIA

## Data Availability

A systematic literature search was conducted in PubMed, MEDLINE, Embase, and Cochrane databases.
